# PageRank Topic Finder based Algorithm for Multimedia Resources in Preschool Education

This article has been retracted.

**DOI:** 10.1155/2022/4173243

**Published:** 2022-07-20

**Authors:** Guiping Yu

**Affiliations:** Normal College, Eastern Liaoning University, Dandong, Liaoning 118000, China

## Abstract

In traditional preschool education, it is time-consuming and laborious to acquire effective materials by using artificial search method. However, with the development of Internet technology, a variety of preschool education institutions or individuals have released their own preschool education resources on the Internet. At present, multimedia technology has been popularized in many schools, and it plays a more and more significant role in teaching. In preschool education teaching, teachers use multimedia resources not only conducive to improve children's learning efficiency but also make the teaching quality from the whole to a higher level. However, some kindergarten teachers rely too much on multimedia in teaching and do not effectively combine it with traditional teaching methods. Sometimes they even use video and related multimedia teaching resources throughout the class, which makes preschool children lack knowledge and knowledge. Therefore, this paper designs a multimedia resource retrieval system based on the theme of preschool education, which mainly achieves the extraction of multimedia resources from web pages and the analysis of multimedia-related text information. In order to design a high-performance topic search algorithm, we must first carry out page parsing, Chinese and English word segmentation, and other page preprocessing. The research results show that it is found that the text-based automatic classification of multimedia resources in preschool education and the filtering of multimedia noise in web pages can provide relevant personnel in the field of preschool education with the retrieval service of multimedia resources.

## 1. Introduction

Traditional teaching methods have many drawbacks. Teachers cannot combine the knowledge they have learned with the real life of young children, but simply and mechanically explain these knowledge points. Grow up healthily and happily. When modern teaching is introduced into the classroom, we can use multimedia's ability to process information such as pictures, colors, language, and sound to form a multimedia teaching system with pictures and texts, which is not only conducive to presenting abstract and difficult knowledge in a more intuitive way, but it can also fully create a lively and pleasant classroom atmosphere, so as to promote children's understanding. When teachers teach new knowledge, children will always encounter some teaching difficulties due to their different thinking development characteristics from adults, and it is difficult to understand this difficult knowledge. At this time, teachers can make good use of multimedia, a new type of teaching equipment, which can not only separate and classify abstract knowledge or incomprehensible concepts in textbooks but also turn this knowledge into vivid pictures. Let the children know at a glance. This not only helps preschoolers remember this difficult knowledge more easily but also helps them to learn actively [1–3]. Based on the above shortcomings, this paper designs and implements an education-oriented multimedia topic searcher. The design of the topic searcher includes two parts: the architecture design and the topic search algorithm design. Among them, the architecture design is the foundation and the topic search algorithm design is the core, and to design a high-performance topic search algorithm, it must first be carried out [4–6]. We must first perform page preprocessing such as page-parsing, Chinese and English word segmentation. At present, the general large-scale search engines have adopted the parallel mechanism, but the improvement effect brought by the parallel is still far from meeting people's needs. People need to improve the current predicament from other angles.

Preschool children are relatively young, their level of understanding is low and their knowledge reserves are small. Therefore, preschool children's education is the beginning of enlightenment education. At this stage, teachers do not need to impart a lot of knowledge to them, but help them establish basic moral concepts and learning simple cultural knowledge are not only conducive to laying a solid foundation for preschool children's future learning but also make it possible to establish correct values and moral values. With the rapid development of information technology, new teaching methods emerge in an endless stream. The previous teaching methods cannot meet the real needs of children, nor can they effectively attract children's attention. Faced with this situation, teachers need to innovate traditional teaching methods and constantly adopt new teaching methods. Multimedia is a new type of teaching equipment under the development of information technology in the new era. It not only integrates sound, picture, audio, animation, and color but also has the advantages of being reproducible, universal, convenient, and fast. Teachers can make full use of this novel equipment to assist teaching, thereby innovating teaching methods. Reasonable application of multimedia teaching in preschool education can activate the classroom atmosphere, and use pictures, words, sounds, and other forms to bring visual and auditory experience to children, and strengthen their understanding of things. It can be seen that discussing multimedia teaching in preschool education and application has certain practical significance [7–9].

Although many preschool educators have integrated multimedia teaching into preschool education, some kindergarten managers only pay attention to multimedia-related equipment, ignoring the training of teachers in related teaching methods in multimedia teaching, even if preschool teachers have conducted relevant training. What they master is only the simple operation of the computer and the related skills of multimedia courseware production. They cannot use other multimedia technology software well and lack multimedia-related teaching methods. Most of these problems are reflected in older kindergarten teachers and township kindergartens with relatively backward economic levels. Some kindergarten teachers lack the understanding of multimedia teaching and do not know the important role of multimedia teaching in early childhood teaching, which affects the application effect of multimedia teaching in preschool education [10–12]. Thematic search engine appears in such a background. Different from general search engines, it mainly provides users with retrieval services of a certain theme or a certain field of resources.

In addition, traditional multimedia teaching is not integrated with traditional teaching resources in terms of resources. Some multimedia teaching resources, such as videos, audios, images, can bring strong sensory stimulation to children. Compared with the traditional teaching mode, they can attract the attention of students and enable teaching activities to be carried out smoothly [13–15]. However, some kindergarten teachers rely too much on multimedia in teaching, and do not effectively combine it with traditional teaching methods. Sometimes they even use videos and related multimedia teaching resources for the whole class, which makes preschool children lack of knowledge and the accumulation a relevant experience. The hands-on operation in the traditional teaching mode cannot be provided by multimedia teaching. Therefore, the single use of multimedia teaching will have a negative impact on the physical and mental development of preschool children [16–18].

Under the current environment, the development of multimedia information retrieval system (as shown in Figure 1) is still in a stage of rapid development, and many companies or scientific research institutions have launched their own related systems. Among these systems, the most representative abroad is the Query By Image Content (QBIC) system designed by IBM, and the Multimedia Information Retrieval System (MIRES) system jointly developed by the Institute of Computing Technology of the Chinese Academy of Sciences and the National Library of China in China.

In the 1990s, in order to realize the commercialization of image retrieval, IBM designed and developed the QBIC image retrieval system, which provides image and dynamic image retrieval services, and is the world's first content-based commercial image retrieval system [19–21]. This system provides a wealth of retrieval methods, and these methods mainly include the following: (1) retrieval using sample images provided by the system; (2) user-designed abbreviated CCTV content of the images to be retrieved or input graphics through other image input devices—retrieval; (3) retrieval by the color or graphic layout of the image; (4) the user inputs that are segments of the moving image or the object in the front and the middle to inquire. When the querier enters the query object (sample image), the system analyzes and extracts the color, line, and structure of the query object in detail, and then processes it according to the retrieval method specified by the querier [22–25]. It should be further explained here that the features used by the system in terms of color include the ratio of various colors, the coordinates of the colors, etc.. The features of lines are based on the improvement of the texture representation method proposed by Tamura, which comprehensively considers the characteristics of granularity, contrast, and texture orientation. In terms of structure, perimeter, area, eccentricity, principal axis deflection and a set of algebraic moment invariants are used. What is even more commendable is that the QBIC system also involves high-dimensional feature indexing, which is rare. The QBIC system is not only based on multimedia content for retrieval but also considers the relationship between text and multimedia resources to a certain extent. For example, for each historical relic in the Palace Museum, it provides accurate and detailed introduction text: age, category, characteristics, the time of admission, and a detailed description of each cultural relic [26, 27].

The structure of this paper is summarized as follows. First, this paper designs a multimedia subject finder for education. Second, the design of topic searcher includes architecture design and topic-search algorithm design. Then, the design of architecture is the base, and the design of topic search algorithm is the core. How to automatically collect these multimedia materials from the vast resource library of the Internet or with as little human participation as possible and automatically classify the collected multimedia materials. In order to solve abovementioned problem, this paper designs a multimedia resource retrieval system based on the theme of preschool education, which mainly achieves the extraction of multimedia resources from web pages and the analysis of multimedia related text information.

In order to design a high-performance topic-search algorithm, we must first carry out page-parsing, Chinese and English word segmentation, and other page preprocessing.

## 2. Topic-Search Algorithm

The topic-search algorithm is the core of the topic searcher, and it is also the key part that distinguishes it from the general searcher; through the preprocessing of the page, various topic information reflecting the topic of the page is extracted. The topic search algorithm is a hot and difficult topic in the study of topic searchers. From the 1990s to the present, many scholars have devoted themselves to this field and have also proposed many search algorithms for practical applications. There are three categories: content-based search algorithms, link structure-based search algorithms, and prior knowledge-based search algorithms.

The basic idea of the search algorithm is summarized as follows: if a page is referenced many times, this page is likely to be important; a page, although not referenced many times, is referenced by an important page, then this page is likely to be important. The importance of a web page is evenly divided and passed on to the pages it links to. The core of the algorithm is the calculation of the PageRank value, and the PageRank value of a page depends on the number of incoming links of the page and the PageRank value of the incoming link page. Suppose the PageRank value of page *p* is PR(*p*), then there is the following iterative formula:

(1) $$\begin{array}{c} \text{PR}\left(p\right)=\frac{\gamma }{T}+\left(1-\gamma \right)\cdot \sum_{r\in in\left(p\right)}\frac{\text{PR}\left(p\right)}{\left|\text{out}\left(r\right)\right|}, \end{array}$$

where *T* is the total number of pages in the calculation, *γ* < 1 is the damping factor, in(*p*) is the set of incoming links for page *p*, and out(*r*) is the set of outgoing links for page *r*. If you want to calculate the PR value of all web pages in the web page set, you must use this formula to iterate repeatedly, and initialize the PR value of each web page to 1/*T*. After a certain number of iterations, the PR value will converge to a relatively fixed value.

The interaction between the central page and the authoritative page can be used for the mining of authoritative pages and the automatic discovery of high-quality Web structures and resources. This is the basic idea of the HITS algorithm. Let the Authority value and Hub value of the page be *A*(*p*) and *H*(*p*), respectively, and the calculation formulas are as follows:

(2) $$\begin{array}{c} A\left(p\right)=\sum_{u\in B\left(p\right)}H\left(u\right),\\ H\left(p\right)=\sum_{u\in F\left(p\right)}A\left(u\right), \end{array}$$

where *B*(*p*) is the set of incoming links of page *p*, and *F*(*p*) is the set of outgoing links of page *p*.

According to the investigation of the distribution of multimedia resources on the Internet, it is found that the links containing multimedia resources have the characteristics of agglomeration, and usually appear in the form of a list of links. These link lists are called “theme groups;” each “theme group” usually has a starting prompt. The text used is called “theme group” title. For example, the “theme group” title that contains multimedia resources may be “excellent courseware,” “multimedia courseware.” Formula (3) is used to express the relevance of link content to a URL link Contributions:

(3) $$\begin{array}{c} \text{Content}\_\text{score}\left(u_{i}\right)=\text{Score}\left(\text{block}\_\text{title}\right)\left[\beta \cdot \text{Score}\left(\text{anchor}\right)+\left(1-\beta \right)\cdot \text{Score}\left(url\right)\right], \end{array}$$

where score is the relevancy between the title of the “topic group” where the link *u*_*i*_ is located and the topic.

In terms of link structure, the link relevancy of parent pages and sibling pages is used to reveal the influence of link structure on the relevancy of a URL link; in order to feedback this influence to each child link in real time, a dynamic factor is introduced to dynamically adjust the degree of influence on each sublink. Equation (4) is used to express the contribution of link structure to the relevance of a URL link:

(4) $$\begin{array}{c} \text{Structure}\_\text{score}\left(u_{i}\right)=\sum_{j=1,u_{i}\in d_{j}}^{t}\frac{\lambda \left(d_{j}\right)P\left(d_{j}\right)}{t}, \end{array}$$

where *u*_*i*_ is the link being crawled, *t* is the total number of parent links, and *λ* is the dynamic factor, calculated with equation (5):

(5) $$\begin{array}{c} \lambda \left(d_{j}\right)=\frac{n^{\prime }+\theta }{n+\theta }, \end{array}$$

where *n*ʹ is the number of topic-related pages in the crawled child links of the parent link *d*_*j*_, *n* represents the total number of crawled child links of the parent link *d*_*j*_, and *θ* is a normalization factor, usually 0.5.

(6) $$\begin{array}{c} P\left(d_{j}\right)=\left(1-\sigma \right)R\left(d_{j}\right)+\sigma \sum_{k=1,d_{k}\in d_{j}}^{N}\frac{P\left(d_{k}\right)}{N}, \end{array}$$

where *σ* is the bias factor, *R* is the topic relevance of parent link *d*_*j*_, *d*_*k*_ is one crawled sublink of *d*_*j*_, and *N* is the total number of crawled sublinks of *d*_*j*_.

When calculating the link relevancy score potential, the two factors of the link content and link structure described above are considered at the same time, which is expressed by formula (7):

(7) $$\begin{array}{c} \text{potential}\_\text{score}\left(u_{i}\right)=\lambda \text{Content}\_\text{score}\left(u_{i}\right)+\left(1-\lambda \right)\text{Structure}\_\text{score}\left(u_{i}\right), \end{array}$$

where *λ* is a scaling factor that balances the weight of link structure and link content. In the standard Fish algorithm, the search width *W* is a fixed value, which is very unreasonable, because the number of links contained in different web pages is very different. Assign a search width *W*_block, use the similarity between the title and the topic of the “topic group” as a coefficient, and operate on it with the following heuristic rule: when a topic-related link is encountered, the *W* value remains unchanged; otherwise, the *W* value decreases by 1; when *W* is 0 or when the “theme group” has finished crawling, enter the next “theme group;” *W* is represented by formula (8):

(8) $$\begin{array}{c} W=\text{Score}\left(\text{block}\_\text{title}\right)\cdot W_{\text{block}}-\rho , \end{array}$$

where *ρ* equals 0 when the topic is relevant; otherwise, *ρ* equals 1.

The premise of automatic classification of documents by a computer is that the computer can “understand” the document. Currently, commonly used classification algorithms generally use a specific model to represent the document. Although multimedia resources can provide intuitive stimulation to human beings and are more acceptable to the public than text, they are more difficult for computers to “understand.” At present, in order to solve this problem, scholars have carried out research work in the following ways: first, use the visual features of multimedia files, such as color, shape, to represent multimedia documents, and its classic application scenario is fingerprint recognition; second, use multimedia-related text content to represent multimedia documents, such as text in flash animation, text next to video in web pages. This method is often used for massive multimedia documents due to its simple operation, low technical difficulty, and good effect—processing. It should be noted that the above two methods are not mutually exclusive and can also be used in combination.

In the vector space model, each document is viewed as a vocabulary set, which is then represented as a vector of term weights:

(9) $$\begin{array}{c} d_{i}=\left(w_{i1},w_{i2},\ldots ,w_{\text{in}}\right), \end{array}$$

where *d* represents a document and *n* represents the dimension of the term space. The weight of each term represents the importance of the term in the document. Usually, we use the TFIDF method or some variant of it to calculate the weights of the terms. The similarity of two documents is represented by the cosine of the angle between their corresponding vectors:

(10) $$\begin{array}{c} Sim\left(d_{i},d_{j}\right)=\frac{\sum_{k=1}^{n}w_{ik}w_{jk}}{\sqrt{\left(\sum_{k=1}^{n}w_{ik}^{2}\right)\left(\sum_{k=1}^{n}w_{jk}^{2}\right)}}. \end{array}$$

When using the space vector model to classify text, the vector is first used to represent the text, which requires the calculation of the weight of the feature item. The TFIDF formula is a commonly used method for calculating the weight of feature items. TFIDF is a statistical method to evaluate the importance of a word or term to a document in a document set or a corpus, that is, to what extent the occurrence of the word can characterize the content of the document. The importance of a word or a term is proportional to the number of times it appears in the document, and the more the number of occurrences of a word or term, the more important it is. Colleagues—the importance of a word or word is inversely proportional to its frequency of different occurrences in the corpus, that is, the more documents a word or word appears in the corpus, the lower the importance of the word or word.

Various forms of TFIDF calculation weights are widely used in retrieval systems. As a measure or rating of the degree of relevance between documents and user queries, the most commonly used TFIDF formula is shown in equation (11):

(11) $$\begin{array}{c} w_{i}\left(d\right)=\frac{tf_{i}\left(d\right)\cdot \;\log\left(N/n_{i}\right)}{\sqrt{\sum_{i}{\left[tf_{i}\left(d\right)\cdot \;\log\left(N/n_{i}\right)\right]}^{2}}}. \end{array}$$

However, it should be noted that except the methods used in the paper, some of the most representative computational intelligence algorithms can be used to solve the problems, such as monarch butterfly optimization (MBO) [28], earthworm optimization algorithm (EWA) [29], elephant herding optimization (EHO) [30], Runge–Kutta optimizer (RUN) [31], and colony predation algorithm (CPA) [32], etc. Then it may perform feature extraction on them and analyze the extracted features.

## 3. System Design and Implementation

As can be seen from Figure 2, although the design details of various topic search engines are different, they are generally composed of the basic parts of topic searcher, indexer, retriever, and user interface. According to needs, you can also add relevant domain knowledge base, user information, resource classifier, and other parts.

A topic searcher is a network resource discovery and collection program, usually starting from a “seed set” (such as user query, seed link, or seed page), requesting and downloading network resources through protocols such as HTTP, analyzing resources and extracting links, and then accessing the network in an iterative manner. The difference between it and the universal searcher is that when the universal searcher selects the next URL to be crawled, it is aimless, and generally uses first-in, first-out (FIFO) order to take out URLs one by one from the URL queue for crawling. This is determined by the goal of general search engines, which are to collect as many pages as possible in a limited time; while the crawling process of topic searchers is target topic driven, it is based on user-defined target topics, from some seeds starting from the URL, follow the hyperlinks on the Web page to traverse the Web online to collect topic-related pages. When traversing, it needs to conduct online analysis, that is, while collecting pages, it judges whether the collected pages are related to the target theme, and sorts the hyperlinks extracted from the pages according to the degree of relevance through a specific algorithm, so that the most relevant it may be that topic-related pages are preferentially crawled. Its overall goal is to collect as many topic-related pages as possible under limited time and space resources, while avoiding topic-irrelevant pages as much as possible.

The function of the indexer is to understand the information searched by the searcher and extract the index items from it to represent the document and generate the index table of the document library. There are two types of index items: objective index items and content index items. Objective index items have nothing to do with the semantic content of documents, such as author name, URL, update time, encoding, length, content index items that are used to reflect the content of documents, such as keywords and their weights, phrases, words. Content index items can be further divided into single index items and multi-index items (or phrase index items). A single-index item is an English word for English, and it is easier to extract, because there are natural separators (spaces) between words; for continuous writing languages such as Chinese, words must be segmented. In a search engine, a weight is generally assigned to a single index item to indicate the degree of discrimination of the index item to the document, and at the same time, it is used to calculate the relevance of the query result. The methods used generally include statistical method, information theory method, and probability method. The extraction methods of multi-index items include statistical method, probability method, and linguistic method. The index table generally uses some form of Inversion List, that is, the corresponding document is searched by the index item. The index table may also record the position where the index item appears in the document, so that the crawler can calculate the adjacent or close relationship (Proximity) between the index items. The indexer can use a centralized indexing algorithm or a distributed indexing algorithm for indexing, and the indexing algorithm has a great impact on the performance of the indexer (such as the response speed during large-scale peak queries). The effectiveness of a search engine depends largely on the quality of the indexer. When the amount of data is large, instant indexing must be implemented; otherwise, it cannot keep up with the rapid increase in the amount of information. Finally, we can build a content-based subject search engine which has strong practical significance both from the perspective of teaching practice and the development of educational technology disciplines.

The retriever quickly retrieves the required resources in the index database according to the user's query, evaluates the similarity between the user's query and the relevant resources in the index database, and then returns it to the user through the user interface according to the similarity. Algorithms, information query, and organization methods will greatly affect the system performance of the retrieval module. There are four commonly used information retrieval models: set theory models, algebraic models, probabilistic models, and mixed models.

This part designs the architecture of multimedia resource retrieval system based on preschool education theme. The system has the following functions: automatic analysis of theme web page grab resource function, classification index function, multimedia resource query function, and background management function.

It can be seen from the functional structure diagram of the system that the multimedia resource retrieval system based on preschool education theme is mainly divided into four subsystems: theme spider, retrieval system, index system, and background service system. These four systems are linked by the database: the theme spider starts to traverse the web pages from the seed website stored in the database, stores the obtained data into the database, and crawls the data source for the system. In the process of parsing the web page, the theme spider automatically filters out those multimedia resources that have nothing to do with the theme, and then uses the text-based method to automatically classify the multimedia, and finally stores the multimedia thumbnails to the server disk, and other related information to the corresponding table in the database. The indexing program uses the inverted index method to process the captured web pages, so as to quickly respond to the user's retrieval requirements. Here we use the open-source component Lucene for indexing. The retrieval subsystem is mainly used to provide a visual interface, and the user is hereafter entering the query keyword, the retrieval subsystem analyzes the user's query requirements, searches the index document for the corresponding information, and feeds it back to the user. The background service mainly includes the following functions: first, manually modify the category of multimedia resources; second, manually modify the category of multimedia resources; delete multimedia noise; third, manually modify other information of multimedia resources; fourth, system-related configuration; fifth, other functions. The idea of background service design is to make up for the insufficiency of the automatic processing program and further improve the accuracy of the system.

According to the previous system function analysis and architecture design, the database entities used in this system are planned. They are seed website entity, web page entity, multimedia resource entity, multimedia resource category entity, feature item entity, and so on.

In this system, the six categories of preschool literature and art, children's health, preschool news, preschool lesson plans, children's entertainment, and educational theory are the author's category planning for preschool education resources under this theme based on the investigation of the current status of the classification of preschool education theme websites. The multimedia resources captured by the system are divided into corresponding categories according to their subject types.

After a total of 105.17 hours of traversing and parsing web pages by the systematic theme spiders, we have acquired about 140,000 multimedia files and their related text description information. Among all the above multimedia resources, the number of different types of multimedia files and their proportions in the total number are shown in Figure 3.

After designing the filtering algorithm, the author selects a certain amount of data from the system database to analyze the algorithm from different angles. The following is the detailed effect analysis. In order to test the filtering effect of the rule-based multimedia noise filtering algorithm on different types of network multimedia files, we randomly selected several multimedia files of each type from the database, and the specific data are shown in Figure 4. The multimedia files listed in the table are all obtained resources without filtering, that is, the system does not know whether they are noise or not.

After processing by the filtering algorithm in the system, the obtained data is shown in Figure 5. The correct rate in the table refers to the ratio of the filtered noise multimedia resources to the total noise multimedia resources. The error rate refers to the proportion of the multimedia resources that mistakenly judge the multimedia resources related to the theme as noise to the total multimedia resources related to the main *P*.

The statistics in the above analysis show that the rule-based multimedia noise filtering algorithm is more accurate in the categories of “children's health,” “preschool news,” “preschool lesson plans” and “children entertainment” than “preschool literature and art,” There are two categories of “children's entertainment.” The reason is that the content of the two categories of “preschool literature and art” and “children's entertainment” is suitable for display in multimedia resources, and the webpages where they are located generally have more multimedia noises, while the other has four categories. The content is rarely displayed in the form of multimedia, that is, occasionally, the number of noisy multimedia in the web page where it is located is also relatively small.

In order to test the effect of noise-like multimedia filtering algorithm in practical application, we randomly arrange a certain 1500 noise-like resources and 1500 nonnoise-like resources. Use the filtering algorithm designed before to judge these resources and obtain the data as shown in Table 1.

According to the data in Table 1, the multimedia noise filter used in this system can filter out 64.0% of the multimedia noise, and the probability that the filter incorrectly judges the subject-related multimedia resources as noise is 27.8%. The above data show that our designed rule-based multivolume noise filter can meet the basic requirements of system operation. In addition, in order to make up for the shortcomings of automatic program processing, we also designed a manual modification module in the background management system to filter out noisy multimedia resources as much as possible and improve the accuracy of the retrieval system. The *x* and *y* variation are shown in Figure 6.

The rule-based multimedia noise-filtering algorithm has achieved certain results in practical applications, but there are still some deficiencies. These deficiencies are embodied in the following two aspects: first, the program execution efficiency is low; second, it cannot filter in the form (size, length, and width) similar to the noise on the subject resource. In response to the above two problems, we have designed the following solutions:

First, strengthen the knowledge of software engineering, optimize the system from the perspective of the overall framework, focus on the preprocessing of multimedia resources, and continuously improve the execution efficiency of algorithm-related programs.

Second, further excavate the meaning of the text related to multimedia resources in the web page, and use the text to interpret the meaning of the multimedia file, and integrate the text information into the rule-based multimedia noise filtering algorithm;

Subsequently, more multimedia files are statistically analyzed to mine the differences between thematic resources and noise resources, thereby improving the accuracy of the algorithm.

Finally, show the program to teachers and classmates, asking them to give guidance and help with revisions. The amplitude is compared in Figures 7 and 8.

The error comparison of the proposed method and LDA is as shown in Figure 9. It can be seen that the proposed method has a lower error.

## 4. Conclusion

This paper designs a multimedia resource retrieval system based on preschool education theme, which mainly realizes the extraction of multimedia resources from web pages and the analysis of multimedia-related text information. The research results show that the text-based automatic classification of preschool education theme multimedia resources and the filtering of multimedia noise in web pages can provide relevant personnel in the field of preschool education with thematic multimedia resource retrieval services.

However, what needs to be explained here is that we only stay on the scientific research conclusions of predecessors and do not conduct more in-depth research on the distribution law of theme pages. How to discover the distribution law of new theme pages and design a new search algorithm, there is still a lot of room for research and exploration.

## Figures and Tables

**Figure 1:** Multimedia information retrieval system.

**Figure 2:** The design details of various topic search engines.

**Figure 3:** Proportions in the total number.

**Figure 4:** The specific data.

**Figure 5:** The obtained data.

**Figure 6:** *x*, *y* variation.

**Figure 7:** Prediction.

**Figure 8:** Amplitude comparison.

**Figure 9:** Error comparison.

**Table 1:** Noise filter filtering results statistics.

Item	Total	Number	Percentage (%)
Filtered noise	1500	691	64
Filtered nonnoise	1500	237	27.8

## Data Availability

The data used to support the findings of this study are available from the author upon request.
